# MiR-96-5p Facilitates Lung Adenocarcinoma Cell Phenotypes by Inhibiting FHL1

**DOI:** 10.1155/2022/7891222

**Published:** 2022-08-16

**Authors:** Feng Zhou, Chaojie Qian, Tingting Chen, Xiaoliang Zang

**Affiliations:** ^1^Department of Respiratory Medicine, Changxing People's Hospital, Huzhou, Zhejiang Province, China 313100; ^2^Department of Respiratory Medicine, The First People's Hospital of Huzhou, Huzhou, Zhejiang Province, China 313000.

## Abstract

**Objective:**

FHL1 is understood as a tumor repressor gene in various cancers and a possible target for cancer treatment. We investigated the influences of FHL1 on cell functions as well as its molecular mechanisms in lung adenocarcinoma (LUAD) cells.

**Methods:**

The miRNA-mRNA modulatory axis was predicted by bioinformatics. The expression levels of FHL1 mRNA and protein in LUAD cells were, respectively, analyzed by qRT-PCR and western blot. Dual luciferase analysis was introduced to verify the interaction between miR-96-5p and FHL1. CCK-8, cell colony formation, and Transwell assays were utilized to analyze proliferation, colony formation, migration, and invasion of A549 cells.

**Results:**

Expression of FHL1 mRNA and protein in LUAD tissue and cells was downregulated, which was linked with poor prognoses of patients. In addition, FHL1 overexpression could hamper colony formation, proliferation, invasion, and migration of LUAD cells. In addition, dual-luciferase analysis verified miR-96-5p as an upstream regulator of FHL1. Overexpression of miR-96-5p suppressed FHL1 expression in LUAD cells and promoted proliferation, invasion, and migration of LUAD cells, while overexpression of FHL1 could simultaneously restore the above-mentioned promoting effect.

**Conclusion:**

MiR-96-5p fostered cell malignant behaviors by targeting FHL1. This research uncovered the regulatory mechanism of FHL1 in LUAD and offered optional therapeutic targets for LUAD patients.

## 1. Introduction

Lung cancer is a type of prevalent malignancy derived from tunica bronchial mucosa or glands. Globally, lung cancer is dominant in cancer morbidity and mortality with its new cases and deaths ranking first among all cancers [1]. The incidence and mortality of lung cancer, one major cause of cancer-related deaths in China, have increased significantly in recent years, with about 7.87 million cases and 631,000 deaths in 2015 [2]. As the predominant type of lung cancer, non-small-cell lung cancer (NSCLC) patients involve 60% of lung adenocarcinoma (LUAD) [3]. LUAD patients in advanced stage are always accompanied with disease metastasis to nearby and distant organs, suggesting their poor prognosis [4]. Hence, an intensive study of LUAD pathogenesis becomes a central issue for seeking out a new target in molecular therapy.

FHL1 is mainly expressed in skeleton and myocardium. FHL1 plays a pivotal role in sarcomere assembly as a scaffold [5], as well as cell cycle and metastasis [6], whose dysfunction is relevant to muscular disorders. FHL1 is considered as a suppressor gene in several tumors. For instance, FHL1 arrests G1/S cell cycle to hamper tongue squamous cell carcinoma cell growth [7]. In glioma, decreased FHL1 protein represses tumor growth via PI3K/AKT signaling transduction [8]. Nevertheless, few investigations have probed into the function of FHL1 in LUAD, which is valuable and ought to be invoked.

MicroRNAs (miRNAs) are capable of affecting tumor formation, cell proliferation, cell invasion, and metastasis via targeting gene expression [9]. Recent investigations have gone deep into aberrantly expressed miRNAs in LUAD. For example, miR-210 targets LOXL4 to facilitate phenotype progression of LUAD [10]. MiR-363-3p constrains LUAD growth via targeting PCNA [11]. MiR-186-5p fosters cell malignant phenotypes of LUAD via PTEN [12]. MiR-96-5p has become a research hotspot in recent years, and it was found to play an essential role in hepatocellular carcinoma [13], gastric adenocarcinoma [14], and head and neck squamous cell carcinoma [15]. Nonetheless, its regulatory role in LUAD has been less well defined.

Herein, we discovered that FHL1 may exert an imperative function in LUAD progression and was a possible target of miR-96-5p. The expression of miR-96-5p was measured by quantitative real-time polymerase chain reaction (qRT-PCR). The mRNA and protein levels of FHL1 in LUAD cell lines were, respectively, analyzed by qRT-PCR and western blot. Through a trail of biological experiments, the effect and modulatory role of miR-96-5p/FHL1 axis in LUAD were authenticated. Together our findings shed novel insights into LUAD development and potential therapeutic approaches.

## 2. Materials and Methods

### 2.1. Bioinformatics Analysis

Mature miRNAs (normal sample: *n* = 46, cancer sample: *n* = 521) and mRNAs (normal sample: *n* = 59, cancer sample: *n* = 535) expression profiles were accessed from The Cancer Genome Atlas (TCGA)-LUAD dataset. Comparison of FHL1 expression between normal and cancer tissue was analyzed by *t*-test. With the medium FHL1 level as threshold, 535 cancer tissue samples were sorted into high- (*n* = 267) and low-expression (*n* = 268) groups. Survival analysis was conducted between the two groups using “Survival” package.

Differential expression analysis was conducted based on miRNAs expression data by “EdgeR” package with |logFC| >2.0 and padj<0.01 as thresholds. miRDB, mirDIP, TargetScan, miRTarBase, and starBase databases were utilized to screen the upstream regulatory miRNAs of FHL1. The overlap miRNAs between the predicted miRNAs and the differentially upregulated miRNAs were considered as the candidates. Pearson correlation analysis was applied to select the most optimal candidate. *t*-test was used to unravel miRNA expression.

### 2.2. Cell Cultivation and Transfection

LUAD cell lines A549 (BNCC100441), H1650 (BNCC232963), H441 (BNCC292357), and H1299 (BNCC334400) and human bronchial epithelial cell line BEAS-2B (BNCC254518) were all procured from BeNa Culture Collection (Beijing, China). Cells were prepared in DMEM or RPMI-1640 medium (Gibco, USA) containing 10% FBS and 100 mg/mL streptomycin/penicillin under routine conditions. The culture conditions were 5% CO_2_ and 37°C. Synthesized miR-96-5p-mimic (miR-mimic), miR-NC, pcDNA3-FHL1 (oe-FHL1), and empty vector pcDNA3 (oe-NC) were all accessed from GenePharma (Shanghai, China). Lipofectamine 2000 Reagent (Invitrogen, USA) was applied for cell transfection. The transfected cells were maintained for 2 d with 5% CO_2_ at 37°C for subsequent experiments.

### 2.3. qRT-PCR

TRIZOL reagent (Thermo Fisher Science, USA) was recommended for total RNA extraction and NanoDrop 2000 spectrophotometer (Thermo Fisher Science, USA) for RNA evaluation and quantification. miScript II RT kit (Qiagen, Germany) as well as PrimeScript RT Master Mix (Takara, Japan) was applied to synthesize complementary DNA (cDNA). Then, miScript SYBR Green PCR Kit (Qiagen, Germany) with SYBR ® Premix Ex Taq TM II (Takara, Japan) was applied to evaluate miRNA and mRNA expression. qRT-PCR was done on Applied Biosystems ® 7500 Real-Time PCR Systems (Thermo Fisher Scientific, USA) to assess miR-96-5p and FHL1 mRNA levels, respectively. U6 and *β*-actin were taken as endogenous references for miR-96-5p and FHL1, respectively. The 2^-*ΔΔ*Ct^ value was utilized to compare relative expression differences. The primer sequences are shown in Table 1.

### 2.4. Western Blot Assay

Following the instructions, protein extraction kit (Beyotime, China) was employed to isolate total proteins. The proteins underwent 10% SDS-PAGE, followed by being transferred onto a PVDF membrane. Then the membrane was blocked with 5% BSA for 1 h and maintained at 4°C with primary antibodies rabbit anti-FHL1 (1 : 1000, ab255828, Abcam, UK) and mouse anti-beta actin (1ug/mL, ab8226, Abcam, UK) overnight. Afterwards, the membrane was incubated for 2 h at room temperature with secondary antibody goat antirabbit IgG H&L (HRP) (1 : 2000, ab6721, Abcam, UK). Thereafter, the membrane was rinsed with PBST three times, and protein level was assayed with ECL kit (GE Healthcare, USA).

### 2.5. Cell Counting Kit-8 (CCK-8) Assay

The transfected cells were placed into 96-well plates (3 × 10^4^ cells/well) for culture. After 10 *μ*L of CCK-8 solution was supplemented at 1, 2, 3, and 4 days of incubation, cells were maintained for 2 h under routine conditions. A microplate reader was employed to assess optical density (OD) value at 450 nm. Based on the OD value, relative growth rate of cancer cells was acquired.

### 2.6. Cell Colony Formation Assay

2 × 10^2^ cells/well were planted on 6-well plates at 37°C for 2 weeks. Following being rinsed with PBS twice, cells were fixed for 5 min with methanol. Then 3 min of cell staining at 37°C was completed with crystal violet. To remove the residual crystal violet, each well was cleaned with sterile water. A microscope was introduced for counting number of colonies (≥50 cells).

### 2.7. Transwell Invasion and Migration Assays

Matrigel (BD Biosciences, USA) was supplemented to upper chamber of Transwell and placed in a humidified incubator for 60 min of gelation at 37°C. LUAD A549 cells were dispersed with trypsin/EDTA (0.25%/0.04%), centrifuged, and washed twice with serum-free culture medium (580 g, 3 min). Then, 2 × 10^5^ transfected cells that suspended in serum-free culture medium were placed on the upper chamber. RPMI-1640 plus 10% FBS was placed below the cell membrane to facilitate cell invasion. 48 h later, cells on the upper layer of the insert with membrane were swabbed with a cotton bud, and cells that invaded through membrane were fixed with 4% paraformaldehyde for 15 min. Next, 25 min of staining at 37°C was done with 0.1% crystal violet. A microscope was used to observe stained cells. The number of stained cells in 5 random fields was counted (100×) for statistical analysis. The experiment was performed in triplicate.

Steps of cell migration assay were the same as cell invasion assay except for addition of Matrigel in invasion assay. The experiment was performed 3 times.

### 2.8. Dual-Luciferase Reporter Gene Assay

Putative targeted relationship between FHL1 and miR-96-5p was predicted through bioinformatics databases. Wild-type FHL1-3′-untranslated region (UTR) sequences (FHL1-WT) and mutant sequences (FHL1-MUT) corresponding to the predicted miR-96-5p binding sites were synthesized and then cloned into dual-luciferase reporter gene vector psiCHECK, respectively. Cells were plated to 24-well plates and prepared in complete culture medium for over 24 h before transfection. PBS (pH 7.4) was employed to rinse cells for transient transfection. The psiCHECK-FHL1 WT/MUT and miR-96-5p mimic/mimic NC were cotransfected with A549 cells with Lipofectamine 2000 (Invitrogen, USA) reagent. Forty-eight h later, cells were harvested, and luciferase activity was assessed and quantified with dual-luciferase reporter assay kit (Promega, USA).

### 2.9. Data Analysis

All data analyses were carried out on GraphPad Prism 6.0 (La Jolla, CA). Each experiment was repeated three times. Data were showed as mean ± SD. *t*-test was utilized for comparison between two groups. *p* < 0.05 suggested statistically significant difference.

## 3. Results

### 3.1. FHL1 Level Is Notably Decreased in LUAD Cells

TCGA-LUAD dataset exhibited that mRNA expression of FHL1 was evidently downregulated in LUAD (Figure 1(a)). Kaplan-Meier analysis revealed that LUAD patients with low FHL1 expression had reduced overall survival (OS) (Figure 1(b)). FHL1 mRNA and protein levels in LUAD cell lines were measured via qRT-PCR and western blot, respectively. As illustrated in Figures 1(c) and 1(d), FHL1 was decreased in A549, H1650, H441, and H1299 cell lines compared with BEAS-2B cell line. Based on previous investigations and experiments, it was authenticated that FHL1 was decreased in LUAD cells. To make a thorough inquiry of the impact of FHL1 on LUAD cells, A549 cell line with the lowest FHL1 expression among all LUAD cell lines was chosen for the subsequent cellular functional experiments.

### 3.2. Overexpression of FHL1 Hinders Cell Malignant Phenotypes of LUAD

To investigate the biological functions of FHL1, we established FHL1 overexpression cell line. Transfection efficiency of FHL1was assayed through qRT-PCR. FHL1 was significantly overexpressed in oe-FHL1 group (Figure 2(a)), thereby being well prepared for following experiments. CCK-8 and cell colony formation experiments exhibited that FHL1 overexpression restrained proliferation and colony formation of A549 cells (Figures 2(b) and 2(c)). Transwell assays showed that FHL1 overexpression in A549 cells repressed the migratory and invasive abilities (Figures 2(d)–2(e)). Taken together, these findings demonstrated that enforced FHL1 level could repress malignant phenotype of LUAD cells.

### 3.3. MiR-96-5p Downregulates FHL1 Level in LUAD Cells

A differential expression analysis was carried out by EdgeR. A total of 112 differential miRNAs were obtained: 92 differentially upregulated miRNAs and 20 differentially downregulated miRNAs (Figure 3(a)). Then, differentially upregulated miRNAs were intersected with the predicted target miRNAs in the database, by which two targets were obtained: miR-105-5p and miR-96-5p (Figure 3(b)). Pearson correlation analysis was performed subsequently to select the miRNA with high negative correlation with FHL1 at expression manner, where miR-96-5p show the highest negative correlation with FHL1 (Figure 3(c)). In addition, bioinformatics analysis showed significantly highly expressed miR-96-5p in tumor tissues (Figure 3(d)). Later, miR-96-5p expression in normal cells and LUAD cells was assayed through qRT-PCR. Result displayed that miR-96-5p was prominently upregulated in LUAD cells (Figure 3(e)), which was in accordance with previous investigations. Thus, miR-96-5p was dramatically inversely associated with FHL1 and may be an upstream regulatory miRNA of FHL1.

Also, starBase database was employed to identify targeted relationship of miR-96-5p and FHL1 (Figure 3(f)). The binding of FHL1 3′-UTR and miR-96-5p was observed. Dual-luciferase analysis indicated that forced expression of miR-96-5p weakened luciferase activity of FHL1-WT, but did not affect that of FHL1-MUT. Hence, miR-96-5p could target FHL1 (Figure 3(g)). Next, qRT-PCR and western blot were performed to assay mRNA and protein levels of FHL1 in transfected cells (Figures 3(h) and 3(i)), respectively. Thus, enforced miR-96-5p level constrained FHL1 level. The findings proved that miR-96-5p could downregulate FHL1 level in LUAD.

### 3.4. MiR-96-5p Facilitates LUAD Cell Phenotype Progression via Suppressing FHL1

To further examine miR-96-5p/FHL1 regulatory axis in LUAD cells, rescue experiments were designed for verification. MiR-NC+oe-NC, miR-mimic+oe-NC, and miR-mimic+oe-FHL1 groups were established to investigate whether overexpression of FHL1 can rescue impact of miR-96-5p overexpression. qRT-PCR and western blot outcomes displayed that compared with miR-NC-oe-NC group, the levels of FHL1 mRNA and protein in miR-mimic+oe-NC group were prominently decreased. Additionally, the levels of FHL1 mRNA and protein in miR-mimic+oe-FHL1 group were significantly higher than those in miR-mimic+oe-NC group (Figure 4(a)). CCK-8 and cell colony formation assays illustrated that enforced expression of miR-96-5p hastened LUAD cell proliferation. Transwell assays exhibited that transfection of overexpression of miR-96-5p increased migratory and invasive capabilities of LUAD cells. Overexpression of FHL1 and miR-96-5p simultaneously weakened facilitating impact of miR-96-5p on cell phenotype progression of LUAD (Figures 4(b)–4(e)).Thus, miR-96-5p facilitated LUAD cell malignant phenotypes via suppressing FHL1.

## 4. Discussion

Accumulating evidence existed that the expression of various mRNAs is decreased in LUAD, such as PRDM16 [16], MFAP4 [17], and VIPR1 [18]. FHL1 as a tumor repressor gene is authenticated to be poorly expressed in varying cancers, containing liver cancer [19], oral cancer [20], head and neck squamous cell carcinoma [21], and breast cancer [22]. We selected FHL1 as the research object to unravel its specific expression. We revealed that FHL1 expression was decreased in LUAD tissue and cells. Besides, decreased FHL1 was associated with dismal outcomes of patients.

Studies existed that silencing FHL1 noticeably fosters the growth of cervical cancer cells [23], and decreased FHL1 also hastens the growth of breast cancer cells [22], indicating that FHL1 exerted an inhibitory effect in several cancers. To validate the impact of FHL1 level on the progression of LUAD cells, FHL1 expression level was upregulated in LUAD cells. A trail of biological experiments displayed that overexpressed FHL1 repressed cell malignant phenotypes of LUAD. Niu et al. [24] found that overexpression of FHL1 restrains LUAD A549 cell growth, which is congruous with our experimental results. The above findings authenticated that FHL1 serves as a tumor repressor in LUAD.

FHL1 has upstream regulatory genes in multiple cancers. MiR-103 targets FHL1 and inversely modulates its expression in NSCLC [25]. In colorectal and liver tumors, miR-410 targets FHL1, and silencing miR-410 increases FHL1 expression [26]. Dual-luciferase analysis validated targeted relationship of FHL1 3′-UTR and miR-96-5p. Existing investigations unraveled that miR-96-5p serves as an oncogene in varying cancer cells. MiR-96-5p targets CAV1 to restrain AKT phosphorylation and its down-stream Cyclin D1 and P70 protein levels, thereby facilitating cancer cell proliferation and migration [27]. Zhao *et al.* [28] unearthed that miR-96-5p enhances cell proliferative ability while hampers cell apoptosis of LUAD via targeting CYLD. As such, overexpression of miR-96-5p exerts a similar promotive impact on papillary thyroid carcinoma cells [29]. This work proved that miR-96-5p was markedly upregulated in LUAD, and upregulation of miR-96-5p resulted in increased cell proliferation, migration, and invasion. Rescue experiments elucidated that enforced expression of FHL1 could reverse promotion impact of miR-96-5p overexpression on LUAD malignant progression. Together the above findings enunciated that miR-96-5p was increased in LUAD cells and decreased FHL1 expression, which also exacerbated LUAD malignant progression.

Overall, this study verified the decreased expression of FHL1 and increased expression of miR-96-5p in LUAD. FHL1 was the target of miR-96-5p. Overexpression of FHL1 restrained proliferation, invasion, and migration of LUAD cells. This study first proposed that miR-96-5p facilitated malignant phenotypes of LUAD cells by targeting FHL1. Besides, the experimental data suggested that FHL1 may be a potential biomarker for drug development. Nevertheless, the interaction between the expression of these two genes in LUAD tissue has not been proved. In the future, we will focus on this direction.

## Figures and Tables

**Figure 1:** FHL1 expression is notably decreased in LUAD cells. (a) Violin plot of FHL1 level in normal group (green; *n* = 59) and tumor group (orange; *n* = 535); (b) survival curves of high-FHL1 (red) and low-FHL1 (blue) groups. Abscissa represents time (year), and ordinate represents survival rate; (c) FHL1 mRNA expression in A549, H1650, H441, H1299, and BEAS-2B cells; (d) FHL1 protein level in cells; ^∗^*p* < 0.05.

**Figure 2:** Overexpression of FHL1 hinders cell phenotype progression of LUAD. (a) FHL1 level in LUAD A549 cells in oe-NC and oe-FHL1; (b) proliferative efficiency of A549 cells in various transfection groups; (c) colony formative capability of A549 cells in various transfection groups; (d and e) migratory and invasive properties of two groups of A549 cells (100×); ^∗^*p* < 0.05.

**Figure 3:** MiR-96-5p downregulates FHL1 expression in LUAD cells. (a) Volcano map of differential miRNAs in normal and tumor groups in TCGA database. Red indicates differentially upregulated miRNAs, and green indicates differentially downregulated miRNAs; (b) Venn diagram of predicted upstream miRNAs of FHL1 and differential miRNAs; (c) Pearson correlation analysis of FHL1 and its predicted upstream miRNAs; (d) violin plot of miR-96-5p expression in normal (green; *n* = 46) and tumor (orange; *n* = 521) tissue; (e) MiR-96-5p level in BEAS-2B and A549, H1650, H441, and H1299 cell lines; (f) diagram of binding of miR-96-5p and FHL1-WT and FHL1-MUT sequences; (g) luciferase activity of A549 cells in treatment groups (miR-NC and miR-mimic); (h) FHL1 mRNA level in A549 cells; (i) FHL1 protein expression in A549 cells; ^∗^*p* < 0.05.

**Figure 4:** MiR-96-5p facilitates cell malignant behaviors via suppressing FHL1. (a) FHL1 mRNA and protein levels in LUAD A549 cells in varying groups; (b) A549 cell proliferative properties in varying groups; (c) cell colony formation of A549 cells in varying groups; (d and e) migratory and invasive abilities of A549 cells in varying groups (100×); ^∗^*p* < 0.05.

**Table 1:** Primer sequences used in qRT-PCR.

Gene	Primer sequences (5′ →3′)
miR-96-5p	F:5′-TCAACTGGTGTCGTGGAGTCGGCAATTCAGTTGAGAGCAAAAA-3′
	R:5′- ACACTCCAGCTGGGTTTGGCACTAGCACATT-3′
U6	F: 5′-CTCGCTTCGGCAGCACATA-3′
	R:5′-CGAATTTGCGTGTCATCCT-3′
FHL1	F: 5′-GAAGTGTGCTGGATGCAAGA-3′
	R: 5′-GGGGGCTTCCTAGCTTTAGA-3′
*β*-Actin	F: 5′-ATCACCATTGGCAATGAGCG-3′
	R: 5′-TTGAAGGTAGTTTCGTGGAT-3′

## Data Availability

The data used to support the findings of this study are included within the article. The data and materials in the current study are available from the corresponding author on reasonable request.
